RETRACTED

# *κ*-Opioid Receptor Agonist U50448H Protects Against Acute Lung Injury in Rats with Cardiopulmonary Bypass via the CAP-NLRP3 Signaling Pathway

**DOI:** 10.1155/2022/2868135

**Published:** 2022-08-18

**Authors:** Guang-Jie Gao, Dan-Dan Song, Long Li, Fan Zhao, Ying-Jie Sun

**Affiliations:** ^1^Department of Anesthesiology, Air Force Hospital of Northern Theater Command of Chinese PLA, Shenyang 110042, China; ^2^Department of Anesthesiology, General Hospital of Northern Theater Command of Chinese PLA, Shenyang 110016, China

## Abstract

**Objective:**

Acute lung injury (ALI) is one of the common and severe complications of cardiopulmonary bypass (CPB), which is the primary cause of death in intensive care units. Nevertheless, there is a lack of effective treatment for ALI secondary to CPB. *κ*-Opioid receptor (KOR) agonists have been demonstrated to improve lung function after pulmonary hypertension. However, its protective role has been barely reported in CPB-induced acute respiratory distress syndrome (ARDS). Therefore, this research focused on the protective effect of a KOR agonist U50448H on ARDS and investigated its potential relationship with the NOD-like receptor family pyrin domain-containing 3 (NLRP3) inflammasome.

**Method:**

Forty-five rats were randomly allocated into Sham, CPB, and U50448 groups (*n* = 15 rats/group). After a CPB model was successfully established in rats, CPB rats were treated with the KOR agonist U50448H. The values of extravascular lung water (EVLW), alveolar-arterial oxygen tension difference (AaDO2), and respiratory index (RI) were examined, and the lung wet/dry (*W*/*D*) weight ratio was also calculated. Western blot (WB) was utilized to measure the expression of MMP-9, GSDMD-C, GSDMD-N, NLRP3, ASC, pro-Caspase-1, pro-IL-1*β*, and *α*7-nAChR. The immunofluorescence assay was performed for examining the expression of ROS, F480, iNOS, CD206, and *α*7-nAChR. Cell apoptosis was detected by the TUNEL assay. ELISA was used to test the level of LPS in serum and the level of MDA, GSH, SOD, TNF-*α*, IL-4, IL-6, IL-18, and IL-1*β* in lung tissues.

**Results:**

It was observed that the administration of U50448H significantly reduced EVLW values and LPS levels in the lung of rats. Meanwhile, U50448H increased AaDO2 values while decreasing RI values. Moreover, the administration of U50448H alleviated the pathological damage caused by ALI secondary to CPB. U50448H repressed ROS release and oxidative stress responses, as well as lowered LPS levels in plasma and MMP-9 expression in the lung of CPB rats. Furthermore, U50448H facilitated the shift of macrophage phenotype to *M*2. In addition, U50448H decreased the activity of the CAP-NLRP3 inflammasome and suppressed pyroptosis in pulmonary cells.

RETRACTED

**Conclusion:**

The KOR agonist U50448H improved lung function and relieved lung injury in CPB rats, accompanied by diminished ROS and MMP-9 levels in lung tissues, promoted macrophage polarization from *M*1 to *M*2, and reduced NLRP3 inflammasome activities. These results indicated U50448H as a promising drug for the treatment of ALI secondary to CPB.

## 1. Introduction

As a severe acute inflammatory disorder of the lung, acute lung injury (ALI) refers to diffuse parenchymal lung damage induced by various direct or indirect factors and acute respiratory dysfunction attributed to increased permeability of alveolar walls and lung capillaries and interstitial and alveolar edema. This disease is mainly characterized by an imbalance in the ventilation/blood flow ratio and a substantial reduction in lung compliance in terms of pathophysiology and is clinically manifested by respiratory distress and progressive hypoxemia. Despite the complex etiology of ALI, tremendous progress has been achieved in research on the pathogenesis of ALI after half a century. Unfortunately, the exact pathogenesis of ALI is not completely elucidated. Additionally, it is generally exhibited in the current studies that the major pathophysiological change of ALI is the uncontrolled inflammatory response that is caused by excessive activation and recruitment of inflammatory cells in the lung and the mutual activation and interaction of numerous inflammatory factors and effector cells. In this context, inhibiting the uncontrolled inflammatory response may be the key strategy for the treatment of ALI.

Moreover, ALI is one of the major complications following cardiac surgery with cardiopulmonary bypass (CPB) [1]. During CPB, the lung is the first affected organ during ischemia, hypoxia, and reperfusion due to aortic block, cardiac arrest, and resuscitation [2]. Almost all CPB patients suffer from varying degrees of postoperative pulmonary decompensation since the lung is the only organ that is not protected by effective cooling in the extracorporeal circulation system [3]. Among these patients, only temporary subclinical symptoms are present in mild cases of lung injury, while acute respiratory distress syndrome (ARDS) is existent in approximately 2% of severe cases, which have a mortality rate of up to 50% [2]. Accordingly, it is imperative to explore effective strategies for preventing and treating CPB-induced lung injury.

*κ*-Opioid receptor (KOR), composed of 380 amino acids, belongs to the G-protein-coupled receptor family [4]. The KOR agonist, U50488H, has been documented to interfere with hippocampal neurological damage and dramatically reduce cognitive impairment after ischemia [5]. U50488H can prevent acetylcholine transport via the KOR-modulated opioid neural system, hence counteracting the reduction in acetylcholine release triggered by mecamylamine, an N-cholinoceptor-blocking medication, and ameliorating learning and memory deficits [6]. Recently, it has been widely confirmed that KOR agonists are associated with cognitive function and related to lung barrier dysfunction due to pulmonary hypertension [7–9]. However, the effect of U50488H on lung injury induced by CPB has not yet been reported adequately, nor have the detailed mechanisms been elucidated.

RETRACTED

The activation and polarization of macrophages are vital for ALI and lung inflammation by mediating the maintenance of immune homeostasis in lung tissues. Damage during ALI can be decreased through macrophage shift from a resting state to an amoebic active state. Macrophages can be polarized into two phenotypes: the classical *M*1 phenotype that displays proinflammatory functions or the alternative *M*2 phenotype that exerts anti-inflammatory effects. Likewise, little is known about the therapeutic function of U50448H in macrophage polarization.

Inflammasomes are macromolecular complexes formed in the cytoplasm of the organism in response to signals from microbial invasion and destruction. NOD-like receptor family pyrin domain-containing 3 (NLRP3) inflammasomes are implicated in a wide range of inflammatory and other injuries in the lung [10], including transfusion-associated ALI, mechanical ventilation-induced lung injury, asthma, tuberculosis, and pulmonary fibrosis [11, 12]. The NLRP3 inflammasome, an extensively studied inflammasome, recruits the adapter protein apoptosis-associated speck-like protein containing a CARD (ASC) upon the activation of its core protein NLRP3, further recruiting and activating pro-Caspase-1, which induces the cleavage of pro-caspase-1 protein to activated caspase-1. Caspase-1 induces the mature activation of the precursors of the proinflammatory cytokines, interleukin (IL)-1*β* and IL-18 [13, 14]. Multiple studies have discovered the involvement of NLRP inflammasomes in the pathological process of ALI and the alleviation of ALI by the inactivation of NLRP inflammasomes [15]. The modulation of inflammasomes may afflict the levels of local inflammatory factors and influence extracorporeal circulation-induced ALI, as the pathogenesis of extracorporeal circulation-induced lung injury shares many similarities to these diseases. However, the precise mechanisms of NLRP3 inflammasomes in ALI secondary to CPB remain poorly identified.

Our previous studies have unveiled that KOR agonists can mitigate intestinal damage [8] and attenuate postoperative cognitive dysfunction [5] following CPB surgery. Nonetheless, there has hitherto been little research on the mechanism by which KORs protect against CPB-induced lung injury. Consequently, this study focused on the promoting role of U50448H on the analgesic effect of conventional opioids and elaborated that U50448H reduced lung injury after CPB, promoted macrophage polarization, and influenced NLRP3 inflammasomes.

RETRACTED

## 2. Materials and Methods

### 2.1. Animals and Animal Groups

Forty-five Sprague-Dawley rats (weighing 350–400 g) were obtained from Laboratory Animal Center at China Medical University (CMU; certificate number: SCXK [Jing] 2019-0001). These rats were housed in the animal facilities of the Laboratory Animal Center of CMU at 22–24°C with a relative humidity of 50 ± 5% and free access to normal diets and water. Then, the rats fasted for 12 h prior to surgery. The entire animal surgery and experiments were ratified by the IACUC of CMU (Approved no. CMU2020423). After two weeks of acclimatization, the rats were randomly arranged into three groups: Sham, CPB, and KOR agonist (*K*) groups (*n* = 15 rats per group). Rats in the Sham group were subjected to intubation and mechanical ventilation in the right femoral artery, and their right internal jugular vein was catheterized without bypass. Rats in the CPB group underwent CPB surgery with the protocol described below. Rats in the KOR group were injected intravenously with U50488H (1.5 mg/kg, D8040, Sigma, St. Louis, MO, USA) before the CPB surgery.

The original calculation of sample size estimated that 100 patients per group would be needed to detect a three-point difference between groups in a two-sided significance test with a power of 0.8 and an alpha error level of 0.05.

The informed consent form was obtained from all patients prior to enrollment in this study. The study protocol was approved by the Ethics Committee of XX hospital (Approval no. FH-JU20200504). All processes conformed to ethical principles for clinical research in the *Declaration of Helsinki*.

In addition, a blank control group was not designed in this study because the Sham group could already adequately serve as a negative control and the blank control could be dispensed with. Based on the late consideration, we believe that there is no significant difference between the Sham group and the negative control group in the current experiments, although we have not conducted the relevant pre-experiments in the early stage.

### 2.2. Establishment of a CPB Rat Model

The CPB rat model was developed as per the previous publications [16, 17]. The rats were anesthetized by the intraperitoneal injection of pentobarbital sodium at 30 mg/kg, fixed in a supine position on the operating table, intubated, and connected to a small animal ventilator and an anesthesia machine. Afterwards, the anesthesia was maintained with 2% isoflurane. Real-time arterial pressure was monitored by inserting a 22G cannula needle into the left femoral artery. In addition, extracorporeal circulation was established by inserting a 22G cannula needle into the caudal artery and an 18G cannula needle into the right jugular vein (with a lateral hole at the head end). After the tubes were connected and secured, intravenous blood was drained into a reservoir and returned. The dose of medication was adjusted based on the blood gas analysis to maintain MAP >60 mmHg, pH within the normal range, the PaCO_2_ range of 35–45 mmHg, and alkali residual (BE) of −3–3 mmol/L. Mechanical ventilation was resumed after the diversion was gradually terminated when the erythrocyte-specific volume (Hct) reached 0.25. Subsequent to the removal of tubes, mechanical ventilation continued. The residual blood in the reservoir was maintained via slow infusion.

RETRACTED

### 2.3. Examination of Alveolar-Arterial Oxygen Tension Difference (AaDO_2_) and Respiratory Index (RI)

A blood gas analyzer (Roche) was utilized to analyze the artery blood gas level, including arterial partial pressure of oxygen (PaO2), base excess, and Hb content, before the CPB surgery and at 0 h, 1 h, and 2 h after the CPB surgery. The derived variables consisted of the arterial-alveolar oxygen tension ratio (a/A), AaDO2, and RI.

### 2.4. The Measurement of the Lung Wet/Dry (*W*/*D*) Weight Ratio and Extra-vascular Lung Water (EVLW)

Subsequently, rats were euthanized with an overdose of sodium pentobarbital through intraperitoneal injection. The final wet lung weight was detected by weighing the excised left lung from rats. Thereafter, the tissues were dried at 60°C for 48 h, followed by the analysis of the lung *W*/*D* weight ratio. Additionally, EVLW was analyzed as reported in a previous publication [18]. In short, lung tissues were homogenized after the addition of equal quantities of distilled water, and then, 50 mL homogenates were centrifuged at 2,000 × *g* for 10 min before 1 h of cultivation at 5°C. The Hb concentration was tested in the supernatant. Arterial blood, tissue homogenates, and supernatants were dried at 80°C for 72 h, followed by the calculation of water content percentages in the samples. Next, the lobe of the right lung was immersed with 10% formalin for further examination. Other lobes of the right lung were frozen for further biochemical detection. After the rats were anesthetized, the neck was depilated and disinfected, and the neck muscles were cut longitudinally with ophthalmic scissors to fully expose the trachea. An inverted *T*-shaped incision was made on the trachea for intubation, and the trachea was slowly injected with prechilled PBS using a 1-mL syringe, washed 2 times (0.8 mL each wash), and flushed 3 times each wash. The recovered fluid was the bronchoalveolar lavage fluid (BALF). The BALF was centrifuged at 1500 r/min and 4°C for 15 min, and the supernatant was aliquoted into Eppendorf (EP) tubes and cryopreserved at −80°C for late use.

RETRACTED

### 2.5. Enzyme-Linked Immunosorbent Assay

The blood of rats was harvested before the surgery and at 0 h, 1 h, and 2 h after the surgery and centrifuged at 1000*g* for 10 min to collect the serum. Then, the level of lipopolysaccharide (LPS) was detected by ELISA. After the euthanasia of rats, the same amount of lung tissues in rats from different groups were prepared into 10% homogenates, which were centrifuged at 1500*g* for 10 min at 4°C. The levels of malondialdehyde (MDA), glutathione (GSH), superoxide dismutase (SOD), tumor necrosis factor-*α* (TNF-*α*), IL-4, IL-6, IL-18, and IL-1*β* were measured in the supernatant by ELISA as per the instructions of corresponding kits.

### 2.6. Hematoxylin-Eosin (*H* & *E*) Staining

Lung tissues from rats were fixed in formaldehyde for 48 h, dehydrated, and cleared. After that, the lung tissues were paraffin-embedded and cut into 4-*μ*m sections. The sections were dewaxed, rehydrated, and stained with hematoxylin for 5 min. Subsequent to rinsing with PBS, the sections were differentiated with hydrochloric acid ethanol, stained with eosin for 1 min, and mounted with neutral resin. At last, the pathological morphology of lung tissues was analyzed under a microscope.

### 2.7. Terminal Deoxynucleotidyl Transferase dUTP Nick End Labeling (TUNEL) Staining

The apoptosis in lung tissues was detected as instructed in the manuals of an in situ apoptosis detection kit (Roche Diagnostics, Mannheim, Germany). The sections (5 *μ*m) of paraffin-embedded lung tissues were dewaxed, permeabilized, reacted with 50 *μ*L TUNEL solution, and warmed in a humid and dark box at 37°C for 60 min. Thereafter, the sections were cultured with 50 *μ*L streptavidin-horseradish peroxidase (HRP) working solution in a dark box for 30 min. Cell nuclei were stained with 4′,6-diamidino-2-phenylindole (DAPI) for fluorescent staining, followed by routine dehydration and fixation. The sections were observed and photographed under the microscope. For each captured picture, the total of nuclei and the number of TUNEL-positive nuclei were counted to calculate the apoptosis rate.

RETRACTED

### 2.8. Immunofluorescence Assay

The levels of inflammatory factors in the BALF supernatant and the serum were detected with corresponding Quantikine™ ELISA kits. Specifically, the samples were prepared by thawing the serum and BALF samples. Afterwards, all reagents were placed at room temperature prior to the experiment, and washing solution, diluent, and standards of different concentrations were prepared as required. Additionally, the microplate was taken out from the sealed bag that had been equilibrated to room temperature.

Paraffin-embedded lung tissues were dewaxed and hydrated, immersed in 3% hydrogen peroxide solution for 15 min, and rinsed with PBS, followed by antigen retrieval with 0.1 M sodium citrate solution. The tissues were blocked with goat serum and incubated at 37°C for 30 min. Next, the sections were separately probed with diluted antibodies against reactive oxygen species (ROS), F480, inducible nitric oxide synthase (iNOS), CD206, and *α*7-nicotinic acetylcholine receptor (*α*7-nAChR) at 4°C overnight. After being rinsed with PBS, the sections were re-probed with fluorescence-labeled secondary antibodies for 30 min at 37°C. Subsequent to PBS rinsing, the sections were subjected to nucleus staining with DAPI and 10 min of incubation at room temperature. Thereafter, the sections were rinsed with PBS, mounted with neutral resin, and analyzed under a fluorescent microscope.

### 2.9. Western Blot (WB)

Lung tissues were homogenized and reacted with radio-immunoprecipitation assay lysis solution (Thermo, 89900) encompassing protease inhibitors on ice for 30 min, followed by the collection of the supernatant. Then, the concentration of the collected proteins was quantified with a bicinchoninic acid kit (Thermo Fisher Scientific Inc.). The same amount of proteins was loaded, separated by sodium dodecyl sulfate-polyacrylamide gel electrophoresis, and then transferred to a polyvinylidene fluoride membrane. After being blocked in skim milk solution, the membrane underwent overnight incubation with diluted primary antibodies against the C terminal of Gasdermin D (GSDMD-C), the N terminal of GSDMD (GSDMD-C), NLRP3, ASC, pro-Caspase-1, pro-IL-1*β*, matrix metallopeptidase-9 (MMP-9), glyceraldehyde-3-phosphate dehydrogenase, and *α*7-nAChR at 4°C. After PBS rinsing, HRP-labelled secondary antibodies were supplemented for 2 h of cultivation with the membrane at room temperature. Proteins were visualized with the electrogenerated chemiluminescence kit on a gel imaging system. Finally, the results were analyzed based on greyscale value using ImageJ.

### 2.10. Statistical Analysis

The findings were demonstrated as mean ± standard deviation and statistically analyzed using SPSS version 11.5 statistical software (SPSS, Chicago, IL, USA). Normally distributed measurement data were expressed as mean ± standard deviation and analyzed using the student's *t*-test when two groups were compared and one-way analysis of variance when multiple groups were compared, followed by the Bonferroni post hoc test. *P* < 0.05 was considered statistically different.

RETRACTED

## 3. Results

### 3.1. The KOR Agonist U50448H Improves the Lung Epithelial Barrier Function and Reduces ALI in CPB Rats

EVLW, one of the pivotal indicators of ALI, is a marker of the fluid in pulmonary interstitial and alveolar spaces [19]. Therefore, EVLW levels were initially analyzed, which showed an obviously higher level of EVLW in rats of the CPB group than in the Sham group (Figure 1(a), *P* < 0.05). Interestingly, U50448H treatment remarkably diminished the level of EVLW in CPB rats. AaDO_2_ and RI were measured by the blood gas analysis to evaluate lung function. As depicted in Figure 1(b), the values of AaDO2 (Figure 1(b), *P* < 0.05) and RI (Figure 1(c), *P* < 0.05) evidently increased at 0 h, 1 h, and 2 h after the CPB in the CPB group compared to the Sham group. Of note, U50488H treatment partially decreased the values of AaDO_2_ and RI at 0 h, 1 h, and 2 h after the CPB surgery (*P* < 0.05). Furthermore, the concentration of LPS in the serum of rats was analyzed using ELISA to determine the change in inflammatory factor levels. The data displayed that serum LPS concentrations were higher in the CPB group than in the Sham group but observably lower in the U50448H group than in the CPB group (Figure 1(d), *P* < 0.05), suggesting that the KOR agonist U50448H might be effective in the treatment of ALI in CPB rats. *H* & *E* staining was adopted to test histological changes in lung tissues from rats, and the results manifested that rats in the CPB group developed substantial lung damage and intra-alveolar congestion/hemorrhage, accompanied by extensive inflammatory cell infiltration. The lung damage was ameliorated in the U50448H group (Figure 1(e), *P* < 0.05).

### 3.2. U50448H Inhibits Pulmonary Oxidative Stress, Reduces Apoptosis in Lung Tissues, and Downregulates MMP-9 Expression in CPB Rats

Moreover, the rat serum was tested for the levels of SOD, MDA, and GSH, which are common indicators of oxidase stress [20]. The concentration of SOD was reduced, and the level of MDA and GSH was elevated in the CPB group compared to the Sham group (Figure 2(a), *P* < 0.05), which was partially nullified by further U50448H treatment (Figure 2(a), *P* < 0.05). Similarly, U50448H treatment also decreased the overactivity of ROS in lung tissues following the CPB surgery (Figure 2(b), *P* < 0.05). In addition, our data also exhibited that apoptosis in pulmonary tissues was blocked in CPB rats by U50448H treatment (Figure 2(c), *P* < 0.05). Finally, MMP-9 is one of the factors related to ALI because it can increase the alveolar-capillary membrane permeability [20]. In our study, the findings presented that U50448H treatment considerably lowered MMP-9 expression in lung tissues, suggesting that U50448H restored the injured lung function (Figure 2(d), *P* < 0.05).

RETRACTED

### 3.3. U50448H Facilitates Lung Macrophage Polarization to M2 Phenotype in CPB Rats

Our study further dissected the regulatory role of U50448H in lung macrophage polarization. Subsequent to the CPB surgery, there were enhancements in the expression of *M*1 macrophage-related biomarkers including TNF-*α* and IL-6 and decreases in the expression of the *M*2 macrophage-related biomarker IL-4 in rats. Conversely, the levels of TNF-*α* and IL-6 were noticeably diminished and the levels of IL-4 were signally augmented by U50448H treatment (Figure 3(a), *P* < 0.05). Concordantly, immunofluorescence assay results revealed that U50448H treatment contributed to reductions in the level of the *M*1 macrophage-related biomarker iNOS and elevations in the level of the *M*2 macrophage-related biomarker CD206 in lung macrophages (Figure 3(b), *P* < 0.05).

### 3.4. U50448H Activates the Cholinergic Anti-inflammatory Pathway (CAP)

We detected the expression of *α*7-nAChR, a key receptor in the CAP [21], to further ascertain whether U50448H activated the CAP. As reflected by the results of the immunofluorescence assay, no striking difference was observed in *α*7-nAChR expression between the Sham group and the CPB group (Figure 4(a), *P* > 0.05). However, U50448H treatment remarkably increased *α*7-nAChR expression (Figure 4(b), *P* < 0.05). In addition, the same trend was obtained by WB that the upregulation of *α*7-nAChR expression was observed under U50448H treatment (Figure 4(b), *P* < 0.05).

### 3.5. U50448H Represses Cell Pyroptosis Induced by the NLRP3/Caspase-1 Signaling Pathway in Lung Tissues

Finally, the relationship between NLRP3/Caspase-1-mediated cell pyroptosis and U50448H was identified in our research. Firstly, WB analyses of pyroptosis indicators manifested that GSDMD-C and GSDMD-N were both upregulated in the CPB group in contrast to the Sham group, suggesting the rupture of the pulmonary cell membrane and the release of proinflammatory factors. It was illustrated that cell pyroptosis occurred during CPB-induced ALI. Moreover, U50448H treatment might prevent lung tissues from cell pyroptosis. Likewise, our findings exhibited dramatic diminishments in the expression of NLRP3, ASC, pro-caspase-1, and pro-IL-1*β* after U50448H treatment (Figure 5(b), *P* < 0.05), the same as the immunofluorescence assay results of ASC and NLRP3 in lung macrophages (Figure 5(c), *P* < 0.05). Meanwhile, conspicuously downregulated IL-1*β* and IL-18 (inflammatory factors) were also measured following U50448H treatment (Figure 5(d), *P* < 0.05).

RETRACTED

## 4. Discussion

ALI is a clinical syndrome characterized by inflammation and increased capillary permeability, which results from a plethora of pathogenic factors, such as infection, trauma, and inhalation of noxious gases. In the United States, nearly 200,000 individuals are admitted to intensive care units annually due to ALI, and 75,000 deaths occur in spite of aggressive and effective treatment. Although reliable statistical data are not available for China, the incidence rate is assumed to be five times higher in China than in the United States because of the high prevalence of infection as well [22, 23]. CPB-induced ALI has emerged as a clinical issue that afflicts the development of cardiac surgery, directly correlates to the success or failure of surgical therapy, and largely impedes the development of cardiac surgery [24].

Current research suggests that ALI is majorly related to several pathophysiological changes, including the hyperactivation of inflammatory cells in the lung, the release of abundant inflammatory mediators, the mutual activation and interaction of a large number of inflammatory factors and effector cells, and uncontrolled inflammatory responses. Mounting studies have elucidated that CPB can stimulate severe systemic inflammatory responses. Abnormal cytokine release has been extensively accepted to be related to the contact of blood components with the artificial surface of the CPB circuit, operative trauma, abnormal shear stress, and ischemia-reperfusion damage during aortic decompression [25, 26]. At present, no effective therapeutic drugs and treatment options have been yet developed for ALI secondary to CPB. Our study identified the alleviatory role of the KOR agonist U50448H in ALI of CPB rats. Specifically, U50448H curtailed lung injury, reduced the expression of inflammatory factors, decreased apoptosis in lung tissues, partially recovered the function of the injured lung, and inhibited cell pyroptosis in the lungs of CPB rats.

The effective control of macrophage activation and differentiation is useful for orchestrating the balance between inflammation and anti-inflammation in lung tissues during ALI. Lung resting macrophages (*M*0) can be polarized into proinflammatory *M*1 phenotype or anti-inflammatory *M*2 phenotype. In the pathogenesis of ALI, resident alveolar macrophages shift toward *M*1 phenotype, thus secreting large amounts of proinflammatory cytokines. At the end of the therapy phase, macrophages can shift from *M*1 to anti-inflammatory *M*2 phenotype, which decreases the inflammatory responses and accelerates lung recovery to repress lung injury. In our study, the data revealed that U50448H curbed the inflammatory response by promoting the transition of macrophages toward *M*2.

RETRACTED

MMP-9 activity was demonstrated to be appreciably increased in a lung injury animal model [27]. In a study on ALI, the degree of lung injury was lower in MMP-9-deficient mice than in wild-type mice [28]. MMP-9 elevates the permeability of the alveolar-capillary basement membrane to cause ALI [29]. The development of CPB is accompanied by the activation of leukocytes-platelet adhesion [30] and release of inflammatory factors, cytokines, ROS, and other adhesion molecules [31]. The cytokines IL-6 and TNF-*α* have been unveiled to be associated with ALI secondary to CPB [32]. Of note, our research exhibited decreases in the levels of MMP-9 and ROS, and these cytokines after U50448H treatment, indicating U50448H as a promising favorable medicine for the treatment of ALI secondary to CPB.

The CAP is an endogenous neuro-feedback pathway that is regulated by the release of ACh from the vagus nerve to the peripheral tissues as the body is exposed to destructive stimuli that trigger inflammatory responses. ACh can bind to the corresponding receptors on the surface of macrophages or other immune cells and exert anti-inflammatory effects via a series of pathophysiological responses within the body. During ALI, elevated ACh activity results in the activation of inflammatory cells, including macrophages and neutrophils, and inhibits the secretion of proinflammatory factors and chemokines related to inflammatory cells such as alveolar macrophages, which, therefore, leads to the attenuation of inflammation and injury in the lung. Intriguingly, the CAP was observed in our study to be activated by U50448H treatment.

Pyroptosis, a cell necrosis form, is manifested by membrane rupture and the release of intracellular proinflammatory contents and can be induced by the spontaneous activation of the NLRP3 inflammasome [33]. As an assembly of NLRP3, ASC, and pro-Caspase-1 with a molecular weight of approximately 700 KDa, the NLRP3 inflammasome is also a cytoplasmic pattern recognition receptor that is expressed in a variety of cells, including monocytes/macrophages, microglia, lymphocytes, neutrophils, and dendritic cells. The *C*-terminus of NLRP3 recognizes different pathogen-associated molecular patterns (PAMPs) and danger-associated molecular patterns (DAMPs) in the cytoplasm, exposes its effector structural domains through its own oligomerization, and recruits ASC. ASC is recruited to convene pro-caspase-1 through the CARD structural domain and co-assemble into NLRP3 inflammasomes. Upon inflammasome activation by stimulation, pro-caspase-1 is cleaved to caspase-1 through self-shearing and activates pro-IL-1*β* and pro-IL-18 to produce mature IL-1*β* and IL-18, thus culminating in inflammatory responses and tissue damage [23, 34]. Our results unraveled that U50448H could downregulate the *C* and *N* terminals of GSDMD, NLRP3, ASC, pro-caspase-1, and pro-IL-1*β*, as well as block cell pyroptosis, indicating the repressive effects of U50448H on NLRP3 inflammasome-induced cell pyroptosis during ALI secondary to CPB. This is probably because NLRP3 can manipulate the production of proinflammatory cytokines, which maintains the accumulation of inflammatory factors to a certain extent by regulating extracorporeal circulation and diminishes the occurrence of inflammatory diseases [35]. The research of Zhou et al. validated that miR-495 attenuates cardiac microvascular endothelial injury and represses inflammatory cells by negatively modulating the expression of the NLRP3 inflammatory signaling pathway and reducing the levels of proinflammatory factors (TNF-a, IL-6, and IL-LP) in alveolar macrophages. This finding suggests that the modulation of NLRP3 can delay the inflammatory response induced by ALI and can be a potential research target for protection against ALI.

RETRACTED

## 5. Conclusion

It was demonstrated in the present study that the KOR agonist U50448H improved lung function, mitigated lung injury, decreased ROS and MMP-9 expression in lung tissues, augmented macrophage polarization from *M*1 to *M*2, and reduced NLRP3 inflammasomes in CPB rats, proposing U50448H as a promising drug for the treatment of ALI secondary to CPB. In the future, more in-depth studies on the mechanisms underlying ALI are warranted to further clarify the mechanisms of action of these biomarkers and targets in the early detection and prevention of lung injury and other diseases.

## Figures and Tables

**Figure 1:** The KOR agonist U50448H alleviates lung injury in CPB rats. Extravascular lung water and AaDO2, RI, water maze, and neurological function scores were used to evaluate postoperative cognitive dysfunction. (a) The results of extravascular lung water; (b) the results of AaDO2; (c) the value of RI; (d) the concentrations of LPS in the rat serum; (e) the result of *H* & *E* staining (scale bar = 50 *μ*m); ^*∗*^*P* < 0.05.

**Figure 2:** The KOR agonist U50448H reduces the levels of ROS and MMP-9 and apoptosis in lung tissues of ALI rats. (a) The ELISA results of GSH, MDA, and SOD levels. (b) The level of ROS detected by the immunofluorescence assay (scale bar = 50 *μ*m); (c) the results of TUNEL staining (scale bar = 50 *μ*m); (d) Western blot analysis of MMP9 expression. ^*∗*^*P* < 0.05 compared to the Sham group; ^#^*P* < 0.05 compared to the CPB group.

RETRACTED

**Figure 3:** The KOR agonist U50448H polarizes macrophages from the M1 phenotype to the M2 phenotype. (a) The ELISA results of TNF-*α*, IL-6, and IL-4 levels in lung tissues; (b) the levels of iNOS and CD206 in the hippocampus detect by the immunofluorescence assay (scale bar = 50 *μ*m). ^*∗*^*P* < 0.05 compared with the Sham group; ^#^*P* < 0.05 compared with the CPB group.

**Figure 4:** The KOR agonist U50448H promotes the activation of the cholinergic anti-inflammatory pathway. (a) The immunofluorescence assay results of *α*7-nAChR expression in lung tissues (scale bar = 50 *μ*m); (b) Western blot results of *α*7-nAChR expression in lung tissues ns which indicated *P* > 0.05; ^*∗*^*P* < 0.05 compared with the CPB group.

**Figure 5:** The KOR agonist U50448H decreases the level of ASC-NLRP3 inflammasomes. (a) Western blot results of GSDMS-C and GSDMS-N expression in lung tissues; (b) Western blot results of NLRP3, ASC, pro-caspase-1, and pro-IL-1*β* expression in lung tissues; (c) immunofluorescence assay results of NLRP3 and ASC proteins in lung macrophages (scale bar = 50 *μ*m); (d) ELISA results of IL-18 and IL-1*β*. ^*∗*^*P* < 0.05 compared with the Sham group; ^#^*P* < 0.05 compared with the CPB group.

## Data Availability

No data were used to support this study.

## Abbreviations

ALI: Acute lung injury
CPB: Cardiopulmonary bypass
ICU: Intensive care unit
KOR: *κ*-Opioid receptor
AaDO2: Alveolar-arterial oxygen pressure difference
WB: Western blot
EVLW: Extravascular lung water
RI: Respiratory index
IACUC: Institutional animal care and use committee
Hb: Hemoglobin
*W*/*D*: Wet-to-dry
PAMPs: Pathogen-associated molecular patterns
DAMPs: Damage-associated molecular patterns.
